# Role of inhibitors of serine peptidases in protecting *Leishmania donovani* against the hydrolytic peptidases of sand fly midgut

This article has been retracted.

**DOI:** 10.1186/s13071-017-2239-9

**Published:** 2017-06-23

**Authors:** Sudha Verma, Sushmita Das, Abhishek Mandal, Md Yousuf Ansari, Sujata Kumari, Rani Mansuri, Ajay Kumar, Ruby Singh, Savita Saini, Kumar Abhishek, Vijay Kumar, Ganesh Chandra Sahoo, Pradeep Das

**Affiliations:** 1 Department of Molecular Biology, Rajendra Memorial Research Institute of Medical Sciences (ICMR), Agamkuan, Patna, Bihar 800007 India; 2 Department of Microbiology, All India Institute of Medical Sciences, Patna, Bihar 801105 India; 3 National Institute of Pharmaceutical Education and Research, Hajipur, Bihar 844101 India; 4 MM College of Pharmacy, Maharishi Markandeshwar University, Mullana, Ambala, 133207 India; 5 Department of Vector Biology, Rajendra Memorial Research Institute of Medical Sciences, (ICMR), Agamkuan, Patna, Bihar 800007 India; 6 Department of Bioinformatics, Rajendra Memorial Research Institute of Medical Sciences (ICMR), Agamkuan, Patna, Bihar 800007 India

**Keywords:** Sand fly midgut, Trypsin, Chymotrypsin, Inhibitor of serine peptidases, Leishmaniasis

## Abstract

**Background:**

In vector-borne diseases such as leishmaniasis, the sand fly midgut is considered to be an important site for vector-parasite interaction. Digestive enzymes including serine peptidases such as trypsin and chymotrypsin, which are secreted in the midgut are one of the obstacles for *Leishmania* in establishing a successful infection. The presence of some natural inhibitors of serine peptidases (ISPs) has recently been reported in *Leishmania*. In the present study, we deciphered the role of these ISPs in the survival of *Leishmania donovani* in the hostile sand fly midgut environment.

**Methods:**

*In silico* and co-immunoprecipitation studies were performed to observe the interaction of *L. donovani* ISPs with trypsin and chymotrypsin. Zymography and in vitro enzyme assays were carried out to observe the inhibitory effect of purified recombinant ISPs of *L. donovani* (rLdISPs) on trypsin, chymotrypsin and the sand fly midgut peptidases. The expression of ISPs in the amastigote to promastigote transition stages were studied by semi-quantitative RT-PCR and Western blot. The role of LdISP on the survival of ISP overexpressed (OE) and ISP knocked down (KD) *Leishmania* parasites inside the sand fly gut was investigated by in vitro and in vivo cell viability assays.

**Results:**

We identified two ecotin-like genes in *L. donovani, LdISP1* and *LdISP2*. *In silico* and co-immunoprecipitation results clearly suggest a strong interaction of LdISP molecules with trypsin and chymotrypsin. Zymography and in vitro enzyme assay confirmed the inhibitory effect of rLdISP on trypsin, chymotrypsin and the sand fly midgut peptidases. The expression of LdISP2 was found to be strongly associated with the amastigote to promastigote phase transition. The activities of the digestive enzymes were found to be significantly reduced in the infected sand flies when compared to uninfected. To our knowledge, our study is the first report showing the possible reduction of chymotrypsin activity in *L. donovani* infected sand flies compared to uninfected. Interestingly, during the early transition stage, substantial killing was observed in ISP2 knocked down (ISP2KD) parasites compared to wild type (WT), whereas ISP1 knocked down (ISP1KD) parasites remained viable. Therefore, our study clearly indicates that LdISP2 is a more effective inhibitor of serine peptidases than LdISP1.

**Conclusion:**

Our results suggest that the lack of ISP2 is detrimental to the parasites during the early transition from amastigotes to promastigotes. Moreover, the results of the present study demonstrated for the first time that LdISP2 has an important role in the inhibition of peptidases and promoting *L. donovani* survival inside the *Phlebotomus argentipes* midgut.

**Electronic supplementary material:**

The online version of this article (doi:10.1186/s13071-017-2239-9) contains supplementary material, which is available to authorized users.

## Background

Leishmaniasis is a vector-borne tropical disease caused by the protozoan parasites of the genus *Leishmania* and transmitted via the bite of the female phlebotomine sand fly [1]. Amongst the different forms of leishmaniasis, visceral leishmaniasis (VL) is the most severe form. In 2014, more than 90% of new cases reported to the WHO occurred in six countries: Brazil, Ethiopia, India, Somalia, South Sudan and Sudan [2]. The life-cycle of *Leishmania donovani*, the causative agent of Indian VL, alternates between an aflagellated amastigote in mammalian macrophages and a flagellated promastigote in the sand fly midgut [3].

The sand fly midgut derived peptidases were found to be involved in various aspects of the vector-parasite relationship [4]. Serine peptidases of the S1A family, like trypsin and chymotrypsin, were reportedly present in dipteran blood-sucking insects like *Phlebotomus papatasi*, *Phlebotomus langeroni*, *Phlebotomus pernicious*, *Phlebotomus orientalis, Phlebotomus schwetzi*, *Phlebotomus argentipes* and *Lutzomyia longipalpis* [4–8]. These digestive peptidases possess the first and most formidable barrier to the parasite survival inside the sand fly midgut [9]. Dostalova et al. [3] described that within the first 6–12 h of infection, most of the *Leishmania* parasites are killed probably due to the effect of such peptidases.

Peptidase inhibitors are present in *Leishmania* spp. for the protection against the proteolytic activities of the peptidases and to regulate their function. Some of the natural inhibitors of serine peptidases (ISP) are reportedly present in different trypanosomatids such as ISP1 (*Trypanosoma brucei brucei*, *Leishmania major*), ISP2 (*Trypanosoma cruzi*, *Trypanosoma brucei rhodesiense*, *L. major*) and ISP3 (*L. major*) [10, 11]. The presence of LdISP has also been recently reported in *L. donovani* [12]. Specifically, ISPs were considered an inhibitor of the S1A family serine peptidases [11], peptidases that are absent in these protozoan parasites. These parasite-derived peptidase inhibitors are known to protect the invading organism from degradation by the host-derived peptidases [11]. Therefore, we hypothesised that these parasite-derived inhibitors might also regulate the activities of hydrolytic serine peptidases inside the sand fly midgut for their survival.

In the present study, we first examine the physiological target of LdISP1 and LdISP2 by showing their interaction as well as their inhibitory properties with trypsin, chymotrypsin and the sand fly midgut peptidases. The expression of LdISP molecules in the amastigote to promastigote transition stages were studied and the role of LdISP molecules on the survival of ISP overexpressed (ISPOE) and ISP knocked down (ISPKD) *Leishmania* parasites inside the sand fly gut was investigated by in vitro and in vivo cell viability assay. Our findings demonstrated that the down-regulation of ISPs led to an increase in protease activity inside the midgut and ultimately affected the parasite survival during the early phase of infection, whereas OE of ISPs in parasites conferred a survival benefit due to inhibition of the midgut peptidases.

## Methods

### Chemical and reagents

All chemicals of analytical grade were purchased from either Sigma-Aldrich (St. Louis, USA), Amresco (Ohio, USA), or USB (Cleveland, USA). Ni^2+^/NTA agarose matrix and gel extraction kits were purchased from Qiagen (Hilden, Germany). Plasmids and restriction enzymes were purchased from Invitrogen (Grand Island, USA) and Fermentas (Waltham, USA). Antibody against trypsin and chymotrypsin were purchased from Gene Tex (Irvine, USA) and Abcam (Cambridge, UK).

### Comparative modelling and protein-protein interaction studies

Homology models of ISPs (ISP1 and ISP2) were generated to investigate the physical contact (*in silico*) between ISPs and trypsin/chymotrypsin. For 3D modelling, the protein sequence of *L. donovani* ISP1 was retrieved from the NCBI protein database [PDB: XP_003859560.1]. ISP2 was sequenced in our laboratory. To identify a suitable template for homology modelling, a Protein Data Bank (PDB) [13] search was performed against the query sequences using the MODELLER 9v3 program Discovery Studio v2.5 (DSv2.5) [14]. Constructed models were refined and validated by CHARMm force field DSv2.5 [15]. The PDB structure of trypsin [PDB: 4I8H] and chymotrypsin [PDB: 1ACB] were retrieved from PDB database [16, 17] and prepared in DSv2.5. The models were further investigated with a Ramachandran plot using PROCHECK [18], an online tool for investigating the stereochemical quality of the protein. The interaction study was performed with the help of GRAMM-X (Web Server v.1.2.0 program) [19]. Protein-protein interaction of the generated complex model was analysed in DSv2.5. The stability of the complex proteins (ISP1-trypsin, ISP2-trypsin, ISP1-chymotrypsin and ISP2-chymotrypsin) were further investigated with the help of molecular dynamics (MD) simulation using Groningen Machine for Chemical Simulations (GROMACS v 4.0.3) package [20]. After simulation, the time evolving coordinates of the system (trajectories) were processed and analysed.

### Maintenance of parasite culture

Promastigotes of *L. donovani* clones, AG83 (MHOM/IN/1983/AG83) were used in all the experiments and grown at 25 °C in 25 cm^2^ flasks in M-199 medium supplemented with 10% FBS [21]. The culture was initiated at ~1 × 10^5^ parasites/ml and grown in a BOD incubator for 4–5 days before sub culturing (late log phase).

### Protein expression and purification

*Leishmania donovani* ISPs genes named *LdISP1* and *LdISP2* were cloned in pET-28a (+) and pET-15b vectors respectively, expressed in *Escherichia coli* and purified by Ni^2+^/NTA affinity column (see Additional file 1 for details).

### Co-immunoprecipitation

The interaction of the purified rLdISPs (rLdISP1 and rLdISP2) with trypsin and chymotrypsin were studied by co-immunoprecipitation assay using Pierce Co-Immunoprecipitation (Co-IP) Kit. Briefly, anti-trypsin and anti-chymotrypsin antibodies were firstly immobilised with amino-link plus coupling resin (10–75 μg of antibody/affinity column) and incubated overnight at 4 °C. The bait protein such as trypsin or chymotrypsin was incubated individually with prey protein, rLdISP1 or rLdISP2 in 1:1 ratio. The mixture of bait and prey proteins (rLdISP1 + trypsin)/(rLdISP2+trypsin) and (rLdISP1 + chymotrypsin)/(rLdISP2 + chymotrypsin) were added to the respective antibody immobilised resin column and incubated overnight for binding at 4 °C. Co-immunoprecipitation complex was then washed with buffer, eluted and run in SDS-PAGE. Non-activated resin bound protein was used as negative control.

### Maintenance of sand fly colonies and isolation of midgut extract

*Phlebotomus argentipes* were maintained in the insectary of Rajendra Memorial Research Institute of Medical Sciences (RMRIMS), Agamkuan, Patna. During the breeding process, the resulting adult sand flies consisting of both males and females were kept starved for 24 to 48 h. They were then fed on anaesthetized rabbit blood for 2 h. Unfed sand flies (both male and female) were screened and provided with 30% sucrose solution to maintain the colony [22]. Fully engorged female sand flies were isolated after blood-feeding (ABF) and kept for 72 h in standard laboratory conditions at 28 °C to 30 °C temperature and 75–80% relative humidity (detail in Additional file 1). Twenty fully fed female sand flies were taken at different time intervals (0, 4, 8, 12, 16, 20, 24, 36, 48, 60 and 72 h) ABF. Simultaneously, for the enzymatic assay, the midgut was isolated from individual sand flies and pooled. For each group, pools of 10 midguts/100 μl of PBS were prepared and stored at -80 °C until use [23].

### Electrophoretic zymography

Detection of the midgut protease activity and their subsequent inhibition by inhibitors including rLdISPs was performed using an overlay zymography technique according to Vinokurov et al. [24] with minor modifications. Midgut extracts (~1 midgut/lane) were run on a native gel and incubated in 50 mM Tris-HCl, buffer, pH -8 supplemented with the following specific protease inhibitors: PMSF (0.5 mM) for all the serine proteases, benzamidine (0.5 mM) for trypsin, TPCK (0.5 mM) for chymotrypsin, rLdISP1 (1 mM) and rLdISP2 (1 mM) for 30 min. The gels were covered by nitrocellulose membrane pre-soaked in the appropriate substrate and incubated at 37 °C for 30 min. The gels were then removed and diazotized. The tryptic and chymotryptic bands were visualised and analysed after colour production.

### Enzymatic assay of trypsin and chymotrypsin

Trypsin and chymotrypsin activities were measured by enzymatic assay in micro titration plates according to Telleria et al. with minor modifications [23]. The concentration of enzymes (0.1 μM) and substrates (200 μM) used were determined experimentally. Sand flies of different experimental conditions were harvested, the midgut was isolated, and lysates were prepared (detail in Additional file 1). The midgut lysate or trypsin/chymotrypsin solution diluted in 100 mM Tris-HCl (pH 8) were either left untreated or treated with rLdISP1 (0.1 nM-10 μM) or rLdISP2 (0.1 nM–1 μM) for 30 min at 4 °C and incubated with their specific chromogenic substrates (BApNA for trypsin and Suc-AAPF-pNA for chymotrypsin). Cleavage of the substrate was monitored continuously for 45 min in an ELISA reader with filter plate at 410 nm, and enzyme activities were determined. Ecotin (0.1 μM) was used as a positive control. The experiments were performed in triplicate and the data expressed as means ± SD from three independent experiments.

### Semi-quantitative RT-PCR

The parasites of different stages during the amastigote to promastigote transformation phase (0 to 72 h) were harvested, and total RNA was extracted using TRIzol reagent (Invitrogen), and cDNA was prepared. Expression of LdISPs was validated using a semi-quantitative RT-PCR method as discussed previously [25]. ISP1 and ISP2 KD and OE *L. donovani* parasites were generated according to Mukherjee et al. (detail in Additional file 1) [26]. Successful knocked down, and overexpression of LdISP1 and LdISP2 genes were also confirmed by semi-quantitative RT-PCR using specific primers for ISP1 and ISP2 (Additional file 1: Table S1). The PCR conditions involved an initial denaturation at 94 °C for 5 min and 24 amplification cycles (94 °C for 60 s, 60 °C for 55 s, and 72 °C for 2 min) followed by a final extension at 72 °C for 7 min. The PCR products were run on 1.5% agarose gel, and the intensity of the bands was quantified using Quantity-one software (Bio-Rad Gel documentation system).

### Western blot

rLdISP1 and rLdISP2 proteins, obtained after the expression and purification were confirmed by Western blot using anti-His primary antibody. Similarly, the co-immunoprecipitate complex of trypsin-rLdISP1/trypsin-rLdISP2 and chymotrypsin-rLdISP1/chymotrypsin-rLdISP2 were confirmed using anti-trypsin, anti-chymotrypsin, anti-ISP1 and anti-ISP2 antibodies. Further, the expression of LdISP1 and LdISP2 during the amastigote to promastigote transforming phase (0 to 72 h) of *L. donovani* was checked at the protein level using anti-ISP1 and anti-ISP2 antibody respectively. KD and OE of ISP1 and ISP2 genes in *L. donovani* parasites were also confirmed at the protein level according to Das et al. [27] using anti-GFP, anti-ISP1 and anti-ISP2 antibodies. α-tubulin was used as an endogenous control in all the experiments.

### Parasite susceptibility assay to the sand fly midgut lysate

To examine the susceptibility of *L. donovani* to the midgut proteases during the amastigote to promastigote transformation, the axenic amastigotes of WT (pLGFPN-vector transfected), ISP1KD, ISP1OE, ISP2KD and ISP2OE parasites were prepared according to Naderer et al. [28]. Axenic amastigote suspension was incubated at 25 °C for different time intervals (0, 4, 8, 12, 16, 20, 24, 36 and 48 h) during transformation to determine the cell viability. Parasite susceptibility assay was performed according to Pimenta et al. [29]. Approximately 10^3^ parasites/ml of each group was exposed to the midgut lysate (single midgut) prepared at the corresponding time points (i.e. at 0, 4, 8, 12, 16, 20, 24, 36 and 48 h ABF) for 2 h at 25 °C. Cell viability was assessed using trypan blue dye exclusion method [30, 31]. The percent control viability was determined from the geometric mean number of the viable parasites over the number of viable parasites in identical aliquots incubated without exposure to the midgut lysate. The experiments were performed in triplicate, and the data were presented as the mean ± SD of three experimental replicates.

### Experimental infection of *P. argentipes*

*Phlebotomus argentipes* sand flies were infected either with WT, ISP1KD, ISP1OE, ISP2KD or ISP2OE axenic amastigotes of *L. donovani* according to Pruzinova et al. [7]. The amastigotes of each group were resuspended in 1 ml of heat inactivated human blood (~1 × 10^6^ parasites/ml) and fed to the sand flies for 2 h through a chick skin membrane according to Kumar et al. [22] at 37 °C. The sand flies were then kept in standard laboratory conditions (at 28–30 °C and 75–80% relative humidity). An equal number of fully engorged female sand flies was separated from each group. Experiments were performed using two pools of 20 sand fly midguts collected at 0, 4, 8, 12, 16, 20, 24, 36, 48, 60 and 72 h ABF. One pool of the isolated midgut was used to determine the enzyme assay. Another pool was used to check the viability of the parasites/midgut. The midgut homogenate was diluted at 1:1 ratio in M199 media and the viability of the parasites/gut was measured using the trypan blue dye exclusion method using haemocytometer [7, 30]. Furthermore, the parasite load was measured in ISP1KD and ISP2KD infected sand flies according to Myskova et al. [31] and indicated as light (< 100 parasites/gut), moderate (100–1000/gut) or heavy infection (> 1000 parasites/gut).

### Morphological analysis of the parasites

To investigate the role of ISP1 in promastigote differentiation, the whole gut of the WT, ISP1KD and ISP1OE infected sand flies were isolated. The morphology of the parasites was determined according to previously published methods [32–35] (detail in Additional file 1).

### Statistical analysis

All the experiments were performed in duplicate or triplicate, and the results were expressed as the mean ± SD. A Student’s *t*-test was performed for statistical analysis using GraphPad Prism software v5.0. An asterisk (*) denotes *P* ≤ 0.05, and a double asterisk (**) denotes *P* ≤ 0.005, and ‘ns’ denotes non-significant as compared to 0 h, untreated controls or WT as applicable.

## Results

### *In silico* interaction of ISPs with trypsin and chymotrypsin

*In silico* interaction of ISPs with trypsin and chymotrypsin were shown by interface analysis and molecular dynamics simulation study. The interface analysis has shown that a total of eight hydrogen bonds were present between ISP1 and trypsin. Out of different interacting amino acid residues, HIS56 of ISP1 was found to strongly involve in interaction with the ASN77 residue of trypsin by forming two H-bonds. The least distance in the interaction was found for trypsin: TRYPSIN:THR29:HN-ISP1:PHE103:O (Fig. 1a. i, Table 1). However, in the case of interaction between ISP2 and trypsin, a total of seven H-bonds were present. In this case, ASN114 of ISP2 strongly interacts with HIS57 residue of trypsin forming two H-bonds each. The least distance in the interaction was found for ISP2:ASN114:HD21-Trypsin: HIS57:NE2 (Fig. 1a. ii, Table 1). On the other hand, GLN39, LEU40 residues of ISP1 interacts with ASN62 of chymotrypsin forming 3 H-bonds (Fig. 2a. i, Table 2). Similarly, in the case of ISP2, GLY10 residue was involved in interaction with ASP33 residue of chymotrypsin forming three H-bonds each. The least distance for the interaction was found for ISP2:LEU13:HN-Chymotrypsin-I:THR26:OG1 (Fig. 2a. ii, Table 2).

**Fig. 1:** *In silico* interaction of ISP1 and ISP2 with trypsin. Homology model of *L. donovani* ISP1 and ISP2 proteins was prepared by MODELLER 9v3 programme DSv2.5. The interaction of ISP1 and ISP2 proteins with trypsin was performed by GRAMM-X (Web Server v.1.2.0 program) software. The ISP1 interaction is shown as ball and stick, whereas ISP2 interaction is represented as a stick. Hydrogen bond interactions were shown as *dotted black lines*. In addition, molecular dynamics simulation method was used to evaluate the interactions between ISPs and trypsin, using software Gromacs v4.0. **a** H-bond interaction of ISP1 and ISP2 with trypsin (i, ii) performed by GRAMM-X. **b** RMSF profile of ISP1-trypsin complex (*red*) (i) and ISP2-trypsin complex (*purple*) (ii). **c** The contact map of ISP1-trypsin complex (i) and ISP2-trypsin complex (ii). **d** Hydrogen bonding profile within ISP1-trypsin atoms and also with water molecules (i) and within ISP2-trypsin atoms and with the water molecules (ii). **e** The solvent accessible surface area for ISP1-trypsin complex (i) and ISP2-trypsin complex (ii). *Abbreviations*: PHE, phenylalanine; TRP, tryptophan; CYS, cysteine; GLN, glutamine; HIS, histidine; GLY, glycine; SER, serine; ILE, isoleucine; THR, threonine; ASN, asparagines; VAL, valine; ARG, arginine; LEU, leucine; TYR, tyrosine; LYS, lysine; ASP, aspartate; PRO, proline; RMSF, Root Mean Square Fluctuation; SASA, the solvent accessible surface area

**Table 1:** Interaction of *L. donovani* ISP1 and ISP2 with trypsin

	Distance	Donor atom	Acceptor atom
ISP1 and trypsin interacting amino acids			
ISP1:PHE103:HN - TRYPSIN:GLY27:O	2.05316	HN	O
ISP1:TRP135:HE1 - TRYPSIN:SER34:O	2.24518	HE1	O
ISP1:CYS136:HG - TRYPSIN:GLY208:O	2.20266	HG	O
ISP1:GLN139:HE22 - TRYPSIN:ILE53:O	2.06784	HE22	O
TRYPSIN:THR29:HN - ISP1:PHE103:O	1.04559	HN	O
TRYPSIN:ASN77:HD21 - ISP1:HIS56:NE2	1.9625	HD21	NE2
TRYPSIN:ASN77:HD22 - ISP1:HIS56:NE2	2.34771	HD22	NE2
TRYPSIN:VAL152:HN - ISP1:HIS96:NE2	2.4941	HN	NE2
ISP2 and trypsin interacting amino acids			
ISP2:ARG65:HH22 - Trypsin:HIS91:O	2.26049	HH22	O
ISP2:THR74:HN - Trypsin:THR149:OG1	2.17454	HN	OG1
ISP2:THR113:HN - Trypsin:SER96:O	2.39979	HN	O
ISP2:ASN114:HD21 - Trypsin:HIS57:NE2	1.13056	HD21	NE2
ISP2:ASN114:HD22 - Trypsin:HIS57:NE2	2.43346	HD22	NE2
ISP2:LEU116:HN - Trypsin:GLY216:O	1.79443	HN	O
Trypsin:TYR94:HH - ISP2:SER112:OG	2.15161	HH	OG

**Fig. 2:** *In silico* interaction of ISP1 and ISP2 with chymotrypsin. Homology model of *L. donovani* ISP1 and ISP2 proteins was prepared by MODELLER 9v3 programme DSv2.5. The interaction of ISP1 and ISP2 proteins with chymotrypsin was performed by GRAMM-X (Web Server v.1.2.0 program) software. The ISP1 interaction was shown as ball and stick, whereas ISP2 interaction was represented as a stick. Hydrogen bond interactions were shown as *dotted black lines*. In addition, molecular dynamics simulation method was used to evaluate the interactions between ISPs and chymotrypsin, using software Gromacs v4.0. ISP1 and ISP2 interaction with chymotrypsin. **a** H-bond interaction of ISP1and ISP2 with chymotrypsin (i, ii) performed by GRAMM-X. **b** RMSF profile of ISP1-chymotrypsin complex (*red*) (i) and ISP2-chymotrypsin complex (*purple*) (ii). **c** The contact map of ISP1-chymotrypsin complex (i) and ISP2-chymotrypsin complex (ii). **d** Hydrogen bonding profile within ISP1-chymotrypsin atoms and also with the water molecules (i) and within ISP2-chymotrypsin atoms and with water molecules (ii). **e** The solvent accessible surface area for ISP1-chymotrypsin complex (i) and ISP2-chymotrypsin complex (ii). *Abbreviations*: PHE, phenylalanine; TRP, tryptophan; CYS, cysteine; GLN, glutamine; HIS, histidine; GLY, glycine; SER, serine; ILE, isoleucine; THR, threonine; ASN, asparagines; VAL, valine; ARG, arginine; LEU, leucine; TYR, tyrosine; LYS, lysine; ASP, aspartate; PRO, proline; RMSF, Root Mean Square Fluctuation; SASA, the solvent accessible surface area

**Table 2:** Interaction of *L. donovani* ISP1 and ISP2 with chymotrypsin

	Distance	Donor atom	Acceptor atom
ISP1 and chymotrypsin interacting amino acids			
Chymotrypsin:ASN62:HD21 - ISP1:GLN39:OE1	2.31963	HD21	OE1
Chymotrypsin:ASN62:HD21 - ISP1:LEU40:O	1.71151	HD21	O
Chymotrypsin:ASN62:HD22 - ISP1:GLN39:OE1	2.4342	HD22	OE1
ISP2 and chymotrypsin interacting amino acids			
ISP2:GLY10:HT1 - Chymotrypsin_I:ASP33:OD1	1.32826	HT1	OD1
ISP2:GLY10:HT2 - Chymotrypsin_I:ASP33:OD1	2.3921	HT2	OD1
ISP2:GLY10:HT3 - Chymotrypsin_I:ASP33:OD1	2.10518	HT3	OD1
ISP2:LYS11:HN - Chymotrypsin_I:PRO30:O	2.39249	HN	O
ISP2:LEU13:HN - Chymotrypsin_I:THR26:OG1	1.18263	HN	OG1
ISP2:LYS37:HZ3 - Chymotrypsin_E:VAL60:O	1.4347	HZ3	O
ISP2:TYR46:HH - Chymotrypsin_E:VAL88:O	2.42993	HH	O
ISP2:ILE139:HN - Chymotrypsin_E:TYR94:O	2.09708	HN	O

Additionally, molecular dynamics (MD) simulation was performed to study the interaction of ISPs (ISP1 and ISP2) with trypsin and chymotrypsin. The interacting complex (ISPs with trypsin and chymotrypsin) was simulated in explicit solvent condition. The Root Mean Square Fluctuation (RMSF) plot of the system depicted the mean fluctuation in the structure (residue) throughout the simulation. The atoms of ISP1-trypsin complex (Fig. 1b. i), ISP2-trypsin complex (Fig. 1b. ii), ISP1-chymotrypsin (Fig. 2b. i), ISP2-chymotrypsin (Fig. 2b. ii) showed flexibility at different loci, encompassing active site residues where the interaction with trypsin and chymotrypsin has been reported in docking study. The distance between all possible amino acid residue pairs and polar contacts between the ISPs-trypsin (Fig. 1c. i, ii) and ISPs-chymotrypsin (Fig. 2c. i, ii) (3D complex) were investigated by analysing two dimension matrix. Further, the interactions were investigated by analysing intramolecular (protein-protein) and intermolecular (protein and water) contacts. The hydrogen bonds formed by the protein atoms (in the complex state) as well as between the protein and water molecules remained constant throughout the simulations (Fig. 1d. i, ii and Fig. 2d. i, ii). Interestingly, the solvent accessible surface area (SASA) of ISPs-trypsin/chymotrypsin complexes depicted a decrease of 10–30 nm.S^-2^.N^-1^ (Fig. 1e. i, ii and Fig. 2e. i, ii). Therefore, MD simulation data depicted the strong interaction of ISP1 and ISP2 with trypsin and chymotrypsin.

### Co-immunoprecipitation studies

To confirm the *in silico* results, we performed co-immunoprecipitation experiments for studying protein-protein interaction. First, *ISP1* and *ISP2* genes of *L. donovani* (*LdISPs*) were successfully cloned, expressed and purified (Additional file 1: Figure S2). The purified proteins (rLdISP1 and rLdISP2) were confirmed through western blot using anti-His antibody (Fig. 3a, b). In co-immunoprecipitation, the different eluted fractions were immunoblotted and probed with anti-trypsin, anti-chymotrypsin antibody as well as with anti-ISP1 and anti-ISP2 antibody. Anti-trypsin and anti-chymotrypsin probed blot showed the presence of trypsin (Fig. 3c, e; Lanes 4–6) and chymotrypsin (Fig. 3d, f; Lanes 4–6) respectively in the eluted fractions. Faint bands of trypsin (Fig. 3c, e; Lane 3) and chymotrypsin (Fig. 3d, f; Lane 3) were also observed in the wash fraction. Anti-ISP1 probed blot showed rLdISP1 protein eluted with trypsin and chymotrypsin (Fig. 3c, d; Lanes 4–6). However, no band corresponding to rLdISP1 was detected in the flow through and wash fraction with trypsin (Fig. 3c; Lanes 2, 3), but a faint band was observed in the wash fraction with chymotrypsin (Fig. 3d; Lane 2). Similarly, anti-ISP2 probed blot showed that rLdISP2 protein was eluted with trypsin and chymotrypsin (Fig. 3e, f; Lanes 4–6). No band corresponding to rLdISP2 was detected in the flow through (Fig. 3e, f; Lane 2). However, a very faint band of rLdISP2 was detected in the wash fraction (Fig. 3e, f; Lane 3). So the *in silico* and co-immunoprecipitation experiments confirmed that both rLdISP1 and rLdISP2 interact with trypsin and chymotrypsin.

**Fig. 3:** In vitro interactions of purified rLdISPs with trypsin and chymotrypsin. *E. coli* (BL-21) expressing the rLdISP1 and rLdISP2 proteins were purified through Ni^2+^/NTA column and confirmed by Western blot using anti-His primary antibody. **a**, **b** Western blot analysis of the expressed rLdISP1 and rLdISP2 proteins in BL-21 cells, respectively: Lane 1: whole cell lysate of cells (no insert); Lane 2: whole cell lysate of the uninduced cells; Lane 3: whole cell lysate of cells induced at 37 °C (0.75 mM IPTG); Lane 4: sup fraction of the induced cells; Lane 5: purified protein of rLdISP1 or rLdISP2. Interaction of rLdISP1 and rLdISP2 with trypsin (**c**, **e**) and chymotrypsin (**d**, **f**) were performed by co-immunoprecipitation. Trypsin or chymotrypsin antibody was bound to the activated resin and incubated with trypsin or chymotrypsin respectively. The immobilized antibody was further incubated individually with rLdISP1 or rLdISP2. Co-immunoprecipitate was collected and analysed by immunoblot, developed separately with anti-trypsin, anti-chymotrypsin, anti-ISP1 and anti-ISP2 antibodies. **c-f** Lane 1: negative control; Lane 2: flow through; Lane 3: wash fraction; Lanes 4–6: elution 1, elution 2, elution 3, respectively; Lane 7: trypsin or chymotrypsin as a positive control; Lane 8: rLdISP1 or rLdISP2 as a positive control

### rLdISP2 showed stronger inhibitory effect on trypsin and chymotrypsin than rLdISP1

In this study, midguts isolated at different time intervals were used to measure the trypsin and chymotrypsin activity (Fig. 4a, b). The activity increased as the time intervals were increased up to 36 h, after that we observed a decrease in the activity at 48, 60 and 72 h maximum trypsin and chymotrypsin activity was observed at 36 h ABF. Therefore, we have used the midgut extract at 36 h ABF to study the inhibitory effect of rLdISPs. The inhibitory effect of rLdISP1 and rLdISP2 on trypsin and chymotrypsin present in the sand fly midgut were analysed through overlay-zymography (Fig. 4c). Significant reduction in trypsin and chymotrypsin activity was observed in the presence of rLdISP2 (Fig. 4c; Lanes 6, 11). However, less remarkable reduction in activity was observed in the presence of rLdISP1 (Fig. 4c; Lanes 5, 10).

**Fig. 4:** Inhibition of trypsin and chymotrypsin activity by rLdISP1 and rLdISP2 proteins. Midguts were isolated from sand fly at different time intervals (0 to 72 h) after rabbit blood-feeding. The enzymatic assay was performed to observe the maximum trypsin (**a**) and chymotrypsin (**b**) activity. **c** Inhibition of the sand fly trypsin and chymotrypsin activity was analysed by zymography. The midgut isolated at 36 h ABF (1 gut/lane) was either left untreated or treated with rLdISP1, rLdLdISP2, benzamidine or TPCK and PMSF. Residual trypsin (Lanes 2–6) and chymotrypsin (Lanes 7–11) activities were measured by using specific chromogenic substrate. **d-g** Inhibition of trypsin and chymotrypsin activity was analysed by enzymatic assay. Bovine trypsin, chymotrypsin and the sand fly midgut extract were either left untreated or treated with rLdISP1 (1–10 μM), rLdISP2 (0.1 μM-1 μM) and ecotin (0.1 μM). The experiments were performed in triplicates, and data are means ± SD from three separate experiments. A Student’s *t*-test was performed for statistical analysis using GraphPad Prism software v5.0. An asterisk (*) denotes *P* ≤ 0.05, double asterisks (**) denote *P* ≤ 0.005, and ‘ns’ denotes non-significant as compared to untreated controls or WT as applicable. *Abbreviations*: T, trypsin; C, chymotrypsin; E, ecotin; G, midgut extract; S, substrate

The inhibitory effect of rLdISP1 and rLdISP2 on trypsin, chymotrypsin and the sand fly midgut proteases was further analysed by enzymatic assay. Trypsin activity was found to be inhibited by ~55% (*P* = 0.0263) and ~99% (*P* = 0.0004) in the presence of 0.1 μM and 1 μM of rLdISP2, respectively (Fig. 4d). However, when we used the sand fly midgut extract the trypsin activity was inhibited by ~62% (*P* = 0.0001) in the presence of 0.1 μM rLdISP2 and ~99.25% (*P* = 0.0024) in the presence of 1 μM of rLdISP2, whereas, ~38% (*P* = 0.0277) reduction in trypsin activity was observed with 10 μM rLdISP1 (Fig. 4e).

Simultaneously, ~58% (*P* = 0.0376) and ~99.5% (*P* = 0.0025) inhibition of chymotrypsin activity were observed in the presence of 0.1 μM and 1 μM of rLdISP2, respectively (Fig. 4f). However, no significant inhibition was observed in the presence of either 1 μM or 10 μM of rLdISP1. Similarly, chymotrypsin activity was reduced by ~65% (*P* = 0.0053) in the presence of 0.1 μM of rLdISP2 and ~99.88% (*P* = 0.0002) in the presence of 1 μM of rLdISP2 when the sand fly midgut extract was used. However, only ~41% (*P* = 0.0361) inhibition of sand fly chymotrypsin activity was observed with 10 μM rLdISP1 (Fig. 4g).

### Differential expression of LdISPs during the amastigote to promastigote phase transformation

No significant expression of LdISP1 was observed during 0 to 8 h. However, from 12 h onwards, a gradual increase in LdISP1 expression was observed. Approximately a 1.7-fold (*P* = 0.0359) and ~2-fold (*P* = 0.0226) increase in LdISP1 expression were observed at 72 h when compared to 12 h at the transcript (Fig. 5a) and protein level (Fig. 5b), respectively. These results indicate that the expression of ISP1 was specific to the promastigote stage only. On the other hand, LdISP2 expression was observed to be differentially regulated during the amastigote to promastigote transformation. The expression of LdISP2 transcript was found to be downregulated by ~2-fold (*P* = 0.0477) at 8 h when compared to 0 h, and ~2.9-fold (*P* = 0.0219) increase in expression was observed at 72 h when compared to 12 h (Fig. 5a). Moreover, the expression of LdISP2 was also found to be upregulated by ~1.8-fold (*P* = 0.019) at 72 h when compared with 12 h at the protein level (Fig. 5b).

**Fig. 5:** Differential expression of LdISP1 and LdISP2 during the amastigote to promastigote transformation of *Leishmania* parasites. The *Leishmania* amastigotes were incubated for 0 to 72 h at 25 °C for their transformation to promastigotes. **a** After the incubation, RNA was isolated by cells pellet and cDNA prepared followed by semiquantitative RT-PCR, α-tubulin PCR was conducted to show uniform expression of a house-keeping gene in all the conditions. The PCR product was run on agarose gel and observed under Gel Doc. Figures represent the relative band intensities of LdISP1 and LdISP2 genes during the transforming phase from 0 to 72 h. **b** After individual incubation, cells were harvested, and proteins were isolated. Western blot was performed to see the expression of LdISP1 and LdISP2 at the protein level by using anti-ISP1 and anti-ISP2 antibodies respectively. Densitometric analysis showed the relative fold increase in the band intensities of LdISP1 and LdISP2 genes expressed in treated parasites when compared to the control (0 h). Experiments were performed in triplicate. Gel and blot images are representative of a single experiment. An asterisk (*) denotes *P* ≤ 0.05, when compared to 0 h

### ISP2 KD parasites are more sensitive to the midgut lysate in comparison to ISP2OE parasites

The role of leishmanial ISPs in the survival of the parasite, inside the sand fly midgut was evaluated. First, ISP1 and ISP2 KD and OE parasites were prepared. KD and OE of ISPs genes in *L. donovani* were confirmed by semi-quantitative RT-PCR and Western blot. An approximate 4-fold decrease (*P* = 0.0222) and ~3-fold increase (*P* = 0.0134) in ISP1 expression were observed in ISP1KD and ISP1OE parasites respectively compared to WT *L. donovani* (Fig. 6a). The expression level of ISP2 was also found to be decreased by ~3-fold (*P* = 0.0241) and increased by ~3.5-fold (*P* = 0.0068) in ISP2KD and ISP2OE parasites, respectively, compared to WT (Fig. 6b).

**Fig. 6:** Knocked down and overexpression of ISP1 and ISP2 genes in *L. donovani*. ISP1 and ISP2 KD and OE constructs were prepared and transfected in *L. donovani*. After successful transfection, RNA was isolated from WT, KD and OE parasites. cDNA was prepared followed by semiquantitative RT-PCR for (**a**) LdISP1 and (**b**) LdISP2, α tubulin was taken as endogenous control. Proteins were extracted from transfected parasites. Down regulation and overexpression of LdISP1 and LdISP2 was further checked at protein level by Western blot by using (**c**) anti-GFP antibody: Lane 1: WT parasites; Lane 2: only pLGFPN vector transfected parasites; Lane 3: ISP2KD parasites; Lane 4: ISP2OE parasites; Lane 5: ISP1KD parasites; Lane 6: ISP1OE parasites (**d**) anti-ISP1 antibody: Lane 1: WT parasites; Lane 2: only pLGFPN transfected parasites; Lane 3: ISP1KD parasites; Lane 4: GFP-tagged ISP1OE parasites. (**e**) anti-ISP2 antibody: Lane 1: WT parasites; Lane 2: only pLGFPN vector transfected parasites; Lane 3: ISP2 KD parasites; Lane 4: GFP-tagged ISP2OE parasites. α tubulin was taken as endogenous control. Densitometric analysis showed the relative fold increase in the band intensities of ISP1KD, ISP1OE and ISP2KD, ISP2OE genes or proteins as compared to WT. Experiments were performed in triplicate. Gel and blot images are representative of the single experiment. An asterisk (*) denotes *P* ≤ 0.05 as compared to WT

The Western blot analysis of the whole cell lysate of ISP1KD, ISP1OE, ISP2KD and ISP2OE parasites with anti-GFP antibody detected the GFP, ISP1-GFP and ISP2-GFP proteins at ~28 kDa, ~44.5 kDa and ~45.5 kDa, respectively, in KD and OE parasites (Fig. 6c). Western blot analysis with anti-ISP1 (Fig. 6d) and anti-ISP2 antibody (Fig. 6e) showed the immunoreactive bands of ~16.5 kDa (LdISP1), ~17.5 kDa (LdISP2), ~44.5 kDa (ISP1-GFP) and ~45.5 kDa (ISP2-GFP). A decreased expression of ISP1 and ISP2 by ~2.9-fold (*P* = 0.0413) and ~3.1-fold (*P* = 0.0113) in ISP1KD and ISP2KD parasites respectively, confirmed the downregulation of ISP1 and ISP2 proteins when compared to WT parasites. An increase in the band intensity of ISP1-GFP and ISP2-GFP proteins by ~1.4-fold (*P* = 0.0413) and ~1.5-fold (*P* = 0.0443), respectively, depicted the overexpression of ISP1 and ISP2 proteins in ISP1OE and ISP2OE parasites when compared to WT.

According to Pimenta et al. [29], the parasites at the transition stage are very susceptible to killing by the digestive enzymes. Therefore, the viability of WT, ISP1KD, ISP1OE, ISP2KD and ISP2OE *L. donovani* parasites (amastigotes, transitional stages and promastigotes) under the exposure of the digestive enzymes of the sand fly midgut were evaluated (Fig. 7). The viability of WT parasites was found to be reduced by ~1.5, ~2.3, ~2.6 and ~2.9-fold at 4, 8, 12 and 16 h, respectively, when compared to 0 h. No significant difference in the viability of the parasites of different groups was observed when compared to the WT parasites at 16 h onwards. Our data strongly suggest that the peptidase level present inside the sand fly midgut during early digestive stages (0 to 16 h) is sufficient to kill the parasites. Furthermore, the viability of ISP2KD parasites was decreased by ~1.3, ~1.3, ~1.4 and ~1.3-fold respectively, at 4, 8, 12 and 16 h when compared to WT (4 h; *P* = 0.0264, 8 h; *P* = 0.0142, 12 h; *P* = 0.0480, 16 h; *P* = 0.0306). On the other hand for ISP2OE parasites, the viability was increased by ~1.1, ~1.2, ~1.2 and ~1.3-fold, respectively, at 4, 8, 12 and 16 h when compared to WT (4 h; *P* = 0.0306, 8 h; *P* = 0.0130, 12 h; *P* = 0.0450,16 h; *P* = 0.0176). However, no significant change in the viability was observed in ISP1KD and ISP1OE parasites when compared to WT. Therefore, this data suggest that ISP2KD parasites were more sensitive to killing by the midgut lysate proteases compared to ISP1KD parasites during early transition stage, whereas ISP2OE parasites could effectively abrogate the proteolytic activities of the midgut proteases.

**Fig. 7:** Sensitivity profiles of ISP1KD, ISP1OE, ISP2KD and ISP2OE parasites after treatment of the sand fly midgut lysate. Axenic amastigotes of WT, ISP1KD, ISP1OE, ISP2KD and ISP2OE *Leishmania* parasites were incubated up to 48 h in BOD incubator (25 °C) for transformation to the promastigotes. At different times of incubation (0, 4, 8, 12, 16, 20, 24, 36 and 48 h), cells were treated (for 2 h) with the gut extract (single blood-fed midgut) isolated at the corresponding period. Percent control viability of the parasites was determined from the geometric mean number of the viable parasite incubated with the midgut proteases over the number of viable parasites in identical aliquots incubated without protease treatment. The experiments were performed in triplicate and data are means ± SD from three separate experiments. An asterisk (*) denotes *P* ≤ 0.05 and ‘ns’ denotes non-significant as compared to WT (Student’s *t*-test)

### ISP2KD *L. donovani* could not effectively inhibit trypsin and chymotrypsin activities inside *P. argentipes* midgut

In the present study, we aimed to investigate the enzyme activities in uninfected, and *L. donovani-*infected sand flies. The activity of trypsin and chymotrypsin was increased with increasing time (up to 36 h) in both uninfected and infected sand flies. The maximum activities were observed at 36 h ABF and after 36 h decrease in activities were observed. Trypsin and chymotrypsin activities were found to be decreased by ~1.47-fold (*P* = 0.0311) and ~1.9-fold (*P* = 0.0299) respectively, at 24 h ABF and ~1.5-fold (*P* = 0.0296) and ~1.4-fold (*P* = 0.0253), respectively, at 36 h ABF in the sand flies infected with the parasite when compared to uninfected one (Fig. 8a, b).

**Fig. 8:** Effect of the parasite infection on the early kinetics of the midgut protease activity. *P. argentipes* flies were fed either on human blood or blood containing WT, ISP1KD, ISP1OE, ISP2KD and ISP2OE *Leishmania* parasites. At various times after blood-feeding the midguts were dissected and assayed for trypsin (**a**, **c**) and chymotrypsin (**b**, **d**) activity by using specific chromogenic substrates. The experiments were performed in triplicate and data are means ± SD from three separate experiments. An asterisk (*) denotes *P* ≤ 0.05 when compared to uninfected or WT as applicable (Student’s *t*-test)

Furthermore, the activities of the proteolytic peptidases at different time interval were also measured in ISP1KD, ISP1OE, ISP2KD, ISP2OE and WT *L. donovani* infected sand flies. Trypsin and chymotrypsin activities were found to be increased by ~1.3 fold (*P* = 0.0354) and ~1.7-fold (*P* = 0.0335), respectively, at 24 h ABF, and ~1.4 fold (*P* = 0.0241) and ~1.5-fold (*P* = 0.0387) respectively, at 36 h ABF in ISP2 KD *Leishmania-*infected sand flies compared to WT-infected sand flies. Simultaneously, trypsin and chymotrypsin activities were found to be decreased by ~1.3-fold (*P* = 0.0496) and ~1.6-fold (*P* = 0.0232), respectively, at 24 h ABF, and ~1.4 fold (*P* = 0.0166) and ~1.7-fold (*P* = 0.0287), respectively, at 36 h ABF in ISP2OE *Leishmania*-infected sand flies compared to WT. However, no significant increase in trypsin and chymotrypsin activities was observed in ISP1KD, and ISP1OE *Leishmania*-infected sand flies (Fig. 8c, d).

### ISP2KD parasites are more susceptible to proteases than ISP1KD parasites inside the sand fly

To study the role of ISPs in *Leishmania* survival inside the sand fly midgut, sand flies were infected with ISP1KD, ISP1OE, ISP2KD, ISP2OE and WT *Leishmania* amastigotes. The viability of the parasites inside the sand fly gut at different time intervals (0 to 72 h) was assessed by counting the parasites in the midgut lysate (Fig. 9a). During the early transition stage, the viability of the WT parasites was found to be decreased by ~1.7, ~1.6, ~1.45 and ~1.3- fold at 4, 8, 12 and 16 h, respectively, when compared to 0 h. However, at the same period (4–16 h) ~3.3, ~4.5, ~3.1 and ~2.6-fold decrease and ~1.3, ~1.37, ~1. and ~1.4-fold increase in the viability were observed for ISP2KD and ISP2OE parasites, respectively, when compared to WT. Therefore, our data suggested a significant difference in the viability of the ISP2KD (4 h; *P* = 0.0463, 8 h; *P* = 0.0374, 12 h; *P* = 0.0264, 16 h; *P* = 0.0395) and ISP2OE (4 h; *P* = 0.0322, 8 h; *P* = 0.0268, 12 h; *P* = 0.0422, 16 h; *P* = 0.0154) parasites when compared to WT at the initial digestive stage (4 to 16 h). Interestingly, after 16 h, an increase in the viability of the parasites was observed for each group of infected parasites. From this data, it can be concluded that ISP2KD parasites are more susceptible to killing by the midgut proteases.

**Fig. 9:** ISPsKD and ISPsOE *L. donovani* parasites survival in *P. argentipes* during the early midgut protease stress. Female *P. argentipes* were infected by feeding on human blood containing either of WT, ISP1KD, ISP1OE, ISP2KD and ISP2OE *Leishmania* parasites (~1 × 10^6^ parasites/ml of human blood) and kept at 25 °C from 0 to 72 h after blood-feeding. **a** The early killing of WT, ISP1KD, ISP1OE, ISP2KD and ISP2OE Ld parasites inside the midgut of the sand fly. Trypan blue assay was used to monitored the viability of the parasites/gut, from the midgut infected with a different group of parasites (~10^6^ amastigotes/ml), dissected at different time interval 0–72 h ABF. The visual examination of the dead and live parasites was determined by counting the parasites in Neubauer chamber of haemocytometer under a light microscope. The value represents the geometric mean of ± SD of 20 sand flies/group. The experiment was performed in triplicate. An asterisk (*) denotes *P* ≤ 0.05 as compared to WT. **b** WT, ISP1KD and ISP2KD infected female sand fly midguts were examined microscopically for infectivity. Intensities of infection were classified into three categories according to their intensity: light (< 100 parasites/gut), moderate (100–1000 parasites/gut) or heavy (> 1000 parasites/gut). Numbers above the bar indicate the number of dissected fully fed female sand flies for each group

The percent infectivity of the sand fly gut infected with ISP1KD and ISP2KD parasites was measured at 24, 48 and 72 h ABF (Fig. 9b). At 24 h post-infection, significant differences were observed between infection rate of WT and ISP2KD parasites viz. WT parasites showed high rate of infection (~74%) with ~50% of heavy infection. In contrast, ISP1KD parasites survived less well as their infection rate was significantly lower (~68%) with ~40% of heavy infection. However, ISP2KD parasites were greatly effected and showed ~48% infection rate with only ~8% of heavy infection. On 48 h ABF, significant differences in heavy infection were also observed between ISP1KD- and ISP2KD-infected parasites which correlate with the infected parasites survival strategies inside the sand fly. Infection rate with ISP1KD parasites was ~65% with ~45% of heavy infection, whereas infection rate with ISP2KD parasite was ~55% with only ~20% of heavy infection. In contrast, WT parasite infection rate was ~80% with ~60% of heavy infection. Simultaneously, on 72 h ABF, 85% infection rate was observed with WT parasites with ~75% of heavy infection. A 70% infection rate was observed with ISP1KD parasites with ~50% of heavy infection whereas, in the case of infection with ISP2KD parasites, the infection rate was ~60% with ~30% of heavy infection. Thus, our findings suggested that the downregulation of ISP2 of the parasite, has a direct effect on the infection rate and survival of the parasite inside the sand fly midgut, where as WT parasites escaped the harsh conditions of the gut.

## Discussion

*Leishmania* promastigotes are confined to the digestive tract of the sand fly and undergo a complex developmental process mainly inside the midgut [36]. Therefore, its survival is severely affected by the sand fly midgut digestive enzymes. It was previously reported that the sand fly midgut expresses an abundance of hydrolytic enzymes such as trypsin and chymotrypsin-like serine peptidases [5, 37, 38]. These enzymes have a direct effect on the parasites [5, 6, 8], especially during the transformation from the amastigote to promastigote [29]. Earlier reports also suggested that the modulation or inhibition of the digestive enzymes by external sources [37, 39, 40] or the parasite itself could provide a direct survival benefit for the parasites inside the sand fly.

Serine peptidases of the parasites and their inhibitors present in the host play an important role in the host-parasite interaction. However, the presence of an inhibitor of serine peptidases is limited to trypanosomes including *Leishmania* spp. [10]. It is reported that ~50–80% of the parasites are killed by trypsin during the early blood meal digestion [29]. Inhibitors of serine peptidases of *L. donovani* (LdISP) inhibit serine proteases of the host instead of their own [12]. However, the importance of these ISPs in parasite survival inside the sand fly midgut, particularly in *P. argentipes* is yet to be elucidated. Therefore, in the present study, we attempted to assess the role of LdISPs in the parasite survival inside *P. argentipes* midgut. So, we characterised LdISP1 and LdISP2 and found that these genes encode proteins with sequence similarities to bacterial ecotin, as it was reported earlier [11].

Yang et al. [41] showed that the interaction of bacterial ecotin with trypsin involves a 50S loop and 80S loop in the primary binding site. The 50S loop comprised LEU-52, HIS-53, ARG-53, whereas, the 80S loop consisted of VAL-81, SER-82, THR-83, MET-94 and MET-85 as interacting amino acids responsible for the strong interaction. In our study, PHE, TRP, CYS, GLN, HIS amino acid residues of LdISP1 and ARG, THR, ASN, LEU, SER residues of ISP2 were inferred to be involved in the interaction with trypsin. The interaction results showed that ISP2 has a higher number of identical amino acids as that of ecotin in comparison to ISP1 participating in the interaction.

Further, Clark et al. [42] showed that the interaction of ecotin with chymotrypsin involves GLN-105, GLU-115, ASP-75, ASN-84 amino acids in the primary binding site and THR-89, SER-91, GLY-94, PHE-95, ARG-135, ASN-137, LEU-140, ARG-139 in the secondary binding site. However, our results revealed that ISP1 and ISP2 interaction with chymotrypsin involved GLN, LEU of LdISP1 and GLY, LYS, LEU, TYRO, ILE of ISP2 amino acids respectively. GLY and LYS of ISP2 were the most frequent amino acids participating in the interaction.

Furthermore, the MD simulation of ISPs-trypsin/chymotrypsin confirms major fluctuations near the active site, which is in congruent with the published report by Kar et al. [43]. The contact points in terms of residue distance predict that both the proteins are interacting at domain interface that may facilitate the opening and closing of the active site pocket for the catalytic activity. A similar technique has also been used by Bhutani et al. [44] where they have shown the protein-protein (DprE1-DprE2) interaction by MD simulation in *Mycobacterium tuberculosis*. The decrease of accessibility is more pronounced for hydrophobic than hydrophilic residues confirming hydrophobic effect as major driving forces within the complex that might be responsible for globular folding of ISPs and trypsin/chymotrypsin, so as to protect the core of the protein from the hydrophilic environment. A similar observation has also been published earlier by Anwar et al. [45] where they have reported that the hydrophobic forces surpass over the hydrophilic forces in the formation of a stable complex between Nbp35 and Cfd1. Therefore, our *in silico* study inferred that the strong interaction persists between LdISPs and trypsin/chymotrypsin.

*In silico* protein-protein interaction was further assessed by co-immunoprecipitation technique. In the present study, we have cloned, expressed and purified rLdISP1 and rLdISP2 proteins. The purified rLdISP1 and rLdISP2 proteins were found to be of molecular weight 19.68 kDa and 20.03 kDa, respectively. In immunoblot analysis, the presence of rLdISP1 and rLdISP2 in the eluted fraction confirmed the co-elution of rLdISP1/rLdISP2 with trypsin and chymotrypsin. These data indicated that the co-elution was solely due to stable interaction and immune complex formation such as trypsin-rLdISP1, trypsin-rLdISP2, chymotrypsin-rLdISP1 and chymotrypsin-rLdISP2 proteins.

The presence of serine peptidases in the sand fly midgut and their inhibition by rLdISPs was confirmed through zymography. The technique of zymography is widely used to identify and characterise the proteolytic activity in the crude extracts of many insects [23, 46]. Our zymography data confirmed the presence of trypsin and chymotrypsin and their relative molecular weight in the midgut of *P. argentipes* as evidenced by Pruzinova et al. [7]. Simultaneously, active bands of serine peptidases were strongly inhibited by trypsin and chymotrypsin specific inhibitor benzamidine and TPCK respectively. The inhibitory effect of purified rLdISP1 and rLdISP2 proteins were further checked against these proteases. We observed that rLdISP2 has a significant inhibitory property on the midgut proteases, compared to rLdISP1. Along with the inhibition assay, zymography also helped us determine the molecular weight of the trypsin and chymotrypsin encoded by *P. argentipes.*

The inhibitory effect of purified rLdISPs on trypsin, chymotrypsin and *P. argentipes* peptidases were also confirmed by an enzymatic assay. Notably, it was found that rLdISP2 had a more inhibitory effect than rLdISP1 over all the proteases. Morrison et al. [32] have shown that although ISP1 and ISP2 of *L. major* were capable of inhibiting *P. papatasi* midgut peptidases, ISP2 was found to be more effective. They observed ~55% and ~100% inhibition of trypsin activity at 0.2 μM and 2 μM of ISP2, respectively. However, they did not find significant inhibition of trypsin activity with ISP1. Our results showed ~62% and ~99% inhibition of trypsin activity and ~58% and ~99.8% inhibition of chymotrypsin activity with 0.1 μM and 1 μM of rLdISP2, respectively. Simultaneously, we did not find any significant inhibition of trypsin and chymotrypsin activity even when tested with 10 μM rLdISP1.

On the other hand, when Morrison et al. [32] studied the inhibitory effect of ISP1 and ISP2 on *P*. *papatasi* gut extract, they observed ~40% inhibition of the peptidase activity at 6.7 μM of ISP1 and 100% inhibition of the midgut peptidase activity at 0.2 μM of ISP2. In our study, the sand fly trypsin activity was found to be inhibited by ~38% at 10 μM of rLdISP1, and ~100% inhibition of the sand fly trypsin activity at 1 μM of rLdISP2. Simultaneously, we observed ~65% and ~100% reduction in chymotrypsin activity at 0.1 μM and 1 μM of rLdISP2, respectively. However, only ~41% inhibitions in chymotrypsin activity were observed even with 10 μM of rLdISP1.

The expression of ISPs during the amastigote to promastigote transformation stage of *L. donovani* showed that the expression of LdISP1 and LdISP2 were significantly altered during the amastigote to promastigote transition. Notably, ISP1 expression was found to be insignificant in the amastigotes stage but significant in the promastigote stage, whereas differential expression of ISP2 was observed and found to be present throughout the transition phase. Therefore, our results also indicated that the parasite differentially regulates the expression of ISP2 to overcome the stress condition generated by proteases present in the host as well as in the vector. However, the role of ISP1 is restricted to the promastigote stage only, reflecting its major role in the sand fly and during the host-parasite early interaction.

Based on the presumptive role of ISPs in the inhibition of the serine proteases, we expected that the silencing and overexpression of these genes would affect the midgut protease activity and hence parasite survival. Antisense and sense cloning are a technique used to down regulate and overexpress the function of any particular gene [26]. In the present study successful knocked down and overexpression of LdISPs was carried out by cloning in a pLGFPN expression vector which was further confirmed by semi-quantitative RT-PCR and Western blot.

The activity of the proteolytic enzymes was reported to be delayed [36, 37] or significantly decreased [11] in *L. major* infected *P. papatasi* explaining the regulation of the gut digestive enzyme activity by the parasites. Borovsky et al. [37] have also reported the reduction of trypsin activity by ~36% inside *P. papatasi* due to *L. donovani* infection. In this study, ISPKD and ISPOE *Leishmania* parasites were used to study the effect of LdISPs proteins on the regulation of the sand fly midgut protease activity. Here, we observed a significant decrease in trypsin and chymotrypsin activity inside the sand fly midgut after *Leishmania* infection. Therefore, it is evident that the parasites are capable of downregulating the protease activity. Furthermore, a significant increase in trypsin and chymotrypsin activities in ISP2KD infected sand fly and a decrease in ISP2OE parasites indicated that ISP2 is the key molecule that downregulates the sand fly midgut protease activity. Therefore, our results are in agreement with the previous report which states that ISP of the parasites might be responsible for the reduction in the enzyme activity [23, 32].

Susceptibility of *Leishmania* to the midgut digestive enzymes is stage specific, and transition stage parasites are highly sensitive to the digestive enzymes of the sand fly [29]. Our in vitro and ex vivo findings suggested that ISP2KD parasites were highly susceptible to killing by the sand fly midgut digestive proteases during the early phase of transition. Simultaneously, no significant differences in the cell viability of ISP1KD parasites were observed when compared to WT during the early transition stage. This could be explained by our finding where consecutive expression of ISP2 gene was observed in all the transforming stages of the parasite, whereas, ISP1 expression was strictly restricted to the promastigote stage. Interestingly, from 16 h onwards, no significant differences in the viability of the ISPKD, ISPOE and WT parasites were observed during transformation. The possible explanation might be that after 24 h, the dense glycocalyx such as lipophosphoglycan (LPG), glycosylated phosphatidyl inositol (GPI) [47, 48] and proteophosphoglycan [49] acquired by the promastigotes protect the parasite from the adverse effect of the hydrolytic enzymes.

In our study, the survival and infection rate of the ISP2KD parasite in *P. argentipes* was found to be severely affected at the early transition stage. In contrast, we found that ISP1KD parasites were able to survive and infect *P. argentipes* as that of WT. Pimenta et al. [29] showed that the peritrophic membrane (PM) could protect parasites against the rapid diffusion of the digestive enzyme during the early phase of infection. However, in *P. argentipes* the PM remained present only for the short period (12 h ABF) [7]. The absence of PM exacerbates lethal condition which exists in the blood-fed midgut. Concurrently, delay in PM formation in *P. argentipes* invalidates the role of PM in preventing the parasite from degradation to the digestive enzymes at the very early transition stage (0 to 12 h). Collectively, all these data strengthen our hypothesis that ISP2 of *L. donovani* have a direct effect on the modulation of the midgut digestive enzymes resulting in the parasite survival inside *P. argentipes.*

In vitro study by Morrison et al. [32] showed the role of *L. major* ISP1 in promastigote differentiation. They observed that overexpression of ISP led to shortening of flagellar length whereas down regulation of ISP1 led to increasing in flagellar length. These might be responsible for the difference in flagellar length and cell body size ratio of the parasites that ultimately affected the promastigotes population. A similar finding was also observed when we infected the sand fly with ISP1KD and ISP1OE parasites. In this study we found that during the late stage of infection with ISP1KD and ISP1OE parasites, all three populations of promastigote (i.e. netomonad, leptomonad and metacyclic) get altered when compared with WT infection.

## Conclusion

Our study indicates that the significant inhibition of serine peptidases by ISP2 is required for the optimal adaptation and survival of *Leishmania donovani* inside *P. argentipes* midgut. At the initial stage of infection, *Leishmania* ISP2 might represent a way in which the parasite defends itself from the midgut serine proteases directed against it. From our study, it was also observed that ISP1, on the other hand, could not significantly inhibit the protease activity present inside the gut of *P. argentipes*, whereas it has an exclusive role in promastigote differentiation.

## Additional file

Additional file 1: Text. Supplementary information. **Table S1.** List of the primers used in the experiments. **Figure S1. **Sequence alignment of ecotin with *L.* *donovani* ISP1 and ISP2. **Figure S2.** Cloning, expression and purification of LdISP1 and LdISP2. **Figure S3.** Measurement of trypsin and chymotrypsin activity in the presence of different concentration of rLdISP1 and rLdISP2. **Figure S4.** Generation of construct for LdISP1 & LdISP2 KD and OE.** Figure S5.** Morphological forms of *L. donovani* promastigote inside *P.* *argentipes* during the late stage of infection. (DOCX 929 kb).

## Abbreviations

ABF: After blood-feeding
BApNA: Nα-benzoyl-*DL*-arginine *p-*nitroanilide
GRAMM: Global range molecular matching
PBS: Phosphate buffer saline
PMSF: Phenyl methyl sulfonyl fluoride
Suc-AAPF-pNA: *N-*succinyl- ala-ala-pro-phe p-nitroanilide
TPCK: Tosyl phenylalanyl chloromethyl ketone
